The article "Potential Pleiotropic Genes and Shared Biological Pathways in Epilepsy and Depression Based on GWAS Summary Statistics" was retracted in 2023. Reasons: signs of a paper mill; compromised peer review; unreliable results or conclusions.

# Potential Pleiotropic Genes and Shared Biological Pathways in Epilepsy and Depression Based on GWAS Summary Statistics

**DOI:** 10.1155/2022/6799285

**Published:** 2022-04-12

**Authors:** Han Lin, Wan-Hui Lin, Feng Lin, Chang-Yun Liu, Chun-Hui Che, Hua-Pin Huang

**Affiliations:** ^1^Department of Neurology, Fujian Medical University Union Hospital, Fuzhou 350001, China; ^2^Intensive Care Unit, Department of Neurology, Fujian Medical University Union Hospital, Fuzhou 350001, China; ^3^Fujian Key Laboratory of Molecular Neurology, Fuzhou 350001, China; ^4^Department of Geriatrics, Fujian Medical University Union Hospital, Fuzhou 350001, China

## Abstract

Current epidemiological and experimental studies have indicated the overlapping genetic foundation of epilepsy and depression. However, the detailed pleiotropic genetic etiology and neurobiological pathways have not been well understood, and there are many variants with underestimated effect on the comorbidity of the two diseases. Utilizing genome-wide association study (GWAS) summary statistics of epilepsy (15,212 cases and 29,677 controls) and depression (170,756 cases and 329,443 controls) from large consortia, we assessed the integrated gene-based association with both diseases by Multimarker Analysis of Genomic Annotation (MAGMA) and Fisher's meta-analysis. On the one hand, shared genes with significantly altered transcripts in Gene Expression Omnibus (GEO) data sets were considered as possible pleiotropic genes. On the other hand, the pathway enrichment analysis was conducted based on the gene lists with nominal significance in the gene-based association test of each disease. We identified a total of two pleiotropic genes (*CD3G* and *SLCO3A1*) with gene expression analysis validated and interpreted twenty-five common biological process supported with literature mining. This study indicates the potentially shared genes associated with both epilepsy and depression based on gene expression, meta-data analysis, and pathway enrichment strategy along with traditional GWAS and provides insights into the possible intersecting pathways that were not previously reported.

## 1. Introduction

Epilepsy is a common neurological disease of worldwide public importance, affecting more than 50 million people globally [1]. As one of its most frequent psychiatric comorbidities, depression appears in approximately 30% of patients with epilepsy [2]. Compared to the general adult population, patients with epilepsy have a higher lifetime prevalence of major depressive disorder (MDD) [3, 4]. Other determinants, such as poor seizure control, epilepsy duration, age, and gender, are also associated with the prevalence of comorbid depression [5]. Comorbid depression leads to unsatisfactory medication adherence, worsens the quality of life, and even increases the risk of death for patients with epilepsy, which is a heavy burden for society and the global public health. Of note, mounting publications have indicated that epilepsy and depression impacted each other bidirectionally, where the risk and severity of one disease were positively associated with the other one. A history of major depression has been observed to increase the risk for newly diagnosed unprovoked seizures in population-based case-control studies [6, 7]. The emotional disturbance of depression in patients with epilepsy could promote their perceived severity and the frequency of seizures, therefore resulting in less chance of seizure recovery [8].

Since the comorbidity of epilepsy and depression and their close correlation were ascertained in numerous studies, researchers started to further interpret these results and seek the underlying neurobiological mechanisms. Genetic variants in brain-derived neurotrophic factor (BDNF) [9, 10], *NTRK2* [11], and *COMT* [12] have been examined as risk loci contributing to the high incidence of depression among patients with epilepsy. *BDNF* Val66Met polymorphism could alter the dendritic trafficking of BDNF messenger ribonucleic acid (mRNA) [13, 14] and the secretion of wild-type BDNF in the CNS [15]. *NTRK2* is a gene encoding tropomyosin receptor kinase B (TrkB), which BDNF binds to with high affinity and then activates. One of the neuropathological alterations of depression in temporal lobe epilepsy (TLE) could be the increase of TrkB expression in the hippocampal area and the changed pattern of calbindin cell loss in dentate gyrus as well as longer apical CB + sprouted fibers projecting into the molecular layer [16]. The involvement of BDNF and TrkB in both pathogenesis of epilepsy and development of its comorbid depression indicates that the dysregulation of the BDNF/TrkB signaling pathway could be one of the shared molecular pathways of these two diseases. Besides, previous studies have highlighted the pathogenic role of the disturbance in neurotransmitters, such as glutamate [17, 18], dopamine [19, 20], 5-hydroxytryptamine (5-HT) [21, 22], and gamma-aminobutyric acid (GABA) [23–25], within epilepsy or depression, respectively. Also, the immune system could be one mechanistic mediator, where IL-1 receptor (IL-1R) signaling was found to be linked to the two diseases [26, 27]. Meanwhile, tumor necrosis factor-*α* (TNF-*α*) was reported to mediate the uptake and release of glutamate by glial cells, which provides evidence for the vital role of the immune system in the coexisting of epilepsy and depression [28]. Despite the lack of further robust evidence, these primary findings have implied the overlap of genetic etiology and biological pathways between epilepsy and depression.

In recent years, GWAS has been started to extend our cognitive medium and bound, yielding a possible shared genetic basis of epilepsy and depression. Through GWAS, the heritability (h2) of epilepsy was estimated at 80%, suggesting that the effect of genetic variation on developing epilepsy is 80% [29]. However, only 30% of this heritability was able to be explained by common variants, the rest of which remains unverified [30]. As for depression, its estimated heritability was 30–40% in the past GWAS [31]. However, the overlap of common genetic variation associated with these two diseases was not yet fully explored, and a large number of risk loci or genes with small effect sizes may be omitted due to the limited sample size of previous genome-wide association studies. Therefore, the availability of GWAS summary statistics is significant to identify pleiotropic genetic etiology in an efficient and time-saving manner.

In the current study, we assessed the genetic relationship and figured out the shared biological pathways based on GWAS summary statistics of epilepsy and depression. Through the gene-based test for GWAS data sets along with meta-analysis, we obtained the possible common disease-associated genes, which were subsequently validated by differentially expressed gene (DEG) analysis for GEO data sets concerning the two diseases. Furthermore, pathway-based analyses were conducted to unveil the shared molecular mechanisms.

The rest of the paper is organized as follows: Section 2 describes the material and methods for the proposed analysis of biological pathways between epilepsy and depression based on meta-analysis and gene expression analysis.  Section 3 provides the results of this study analysis. Discussion on these results and previous studies is given in Section 4.  Section 5 concludes this paper.

## 2. Materials and Methods

### 2.1. Data Sources

GWAS summary data were obtained from previously published studies by three international consortia, the International League Against Epilepsy (ILAE) Consortium, the Psychiatric Genomics Consortium (PGC), and the United Kingdom Biobank (UKB). Overlapping samples have been excluded prior to analysis. The analysis flowchart of the total statistics of epilepsy and depression is shown in Figure 1 for a quick glance, where MAGMA is applied to the gene-based analysis of GWAS data of both epilepsy and depression, and the Fisher method is used for the calculation of the combined *P* value.

The epilepsy statistics data were summarized from a genome-wide mega-analysis by the ILAE Consortium on complex epilepsies [32], involving 15,212 cases and 29,677 controls with 4,880,492 quality-controlled single-nucleotide polymorphisms (SNPs) analyzed. The meta-analysis focused on the association of the genetic variants with not only epilepsy of broad phenotype but also specific syndromes or subtypes of epilepsy (i.e., focal epilepsy, generalized epilepsy, and juvenile myoclonic epilepsy). Over 95% of all cases were Caucasian, and the rest were Asian and African. The analysis was conducted after ethnic stratification. We selected the GWAS summary statistics on the epilepsy of broad phenotype for further gene-based study.

The depression GWAS summary statistics which is selected from a large-scale meta-analysis contains 170,756 cases and 329,443 controls [33]. It included the 33 cohorts of PGC and UKB participants described in the previous studies [34, 35]. All samples in both consortia were of European ancestry. A total of quality-controlled 8,483,301 SNPs were imputed. To minimize the possible omission, the phenotype of depression in the UKB cohort was expanded to broad depression based on self-reported help-seeking behaviors, though the phenotype in the PGC study was limited to MDD.

### 2.2. Gene-Based Test Using MAGMA

MAGMA software (version 1.08) was applied to the gene-based analysis of GWAS data using the summary SNP *P* values from the GWAS summary statistics described above [36]. It aggregated the joint associations of multiple SNPs within whole gene areas with depression or epilepsy, giving consideration to the linkage disequilibrium (LD) between SNPs. Compared to pathway scoring algorithm (Pascal) and versatile gene-based association study software (VEGAS), MAGMA computes the statistics results more efficiently with multiple linear regression rather than chi-squared statistics or assignment of simulations to genetic markers [37, 38]. The resulting gene *P* value was calculated based on the SNP-wise mean model to estimate gene associations. Taking into consideration the vital regulatory function of peripheral genes with smaller effects in depression and epilepsy, a *P* < 0.05 was considered statistically significant and defined as a threshold, and genes with this threshold were chosen for subsequent analysis.

### 2.3. Meta-Analysis for GWAS Data

There are many methods available in the literature, such as Edgington's method, Fisher's method, George's method, and Stouffer's method, for combining *P* value. We employed Fisher's method as it is one of the most commonly used meta-analysis approaches, which outperforms for large statistics and is sensitive to the smallest value of P, to calculate the combined *P* value for the gene-based test results of depression and epilepsy GWAS data. The formula is as follows:

(1) $$\begin{array}{c} X^{2}=-2\overset{k}{\underset{i=1}{\sum }}\text{log}\left(p_{i}\right). \end{array}$$

In equation (1), *P*_*i*_ refers to the *P* value of each gene for the *i*th study, and *k* is defined as the total counts of studies. The distribution of statistics is chi-squared, with 2*k* degrees of freedom [39]. Adjusted *P* values by Bonferroni correction were used to reduce type I error. Therefore, *P*_combined_ is considered to be statistically significant when it is less than 0.05/2*N* (*N* is the number of shared genes of depression and epilepsy with *P* < 0.05 in gene-based test). Fisher's method was conducted in R software (version 3.6.2).

### 2.4. Gene Expression Analysis

We searched the GEO database for expression profiles to verify the shared disease-associated genes differentially expressed between patients and healthy controls [40]. The transcriptional regulation of both brain tissue and peripheral blood was accessed between patients with epilepsy or depression and controls.

For epilepsy, we selected data sets of GSE134697, GSE140393, and GSE143272 for differentially expressed gene (DEG) analysis. GEO series GSE143272 detected transcriptome of peripheral blood samples from 91 patients with epilepsy and 50 healthy subjects, which were tested on the Illumina HumanHT-12 V4.0 Expression BeadChip [41, 42]. Temporal lobe epilepsy (TLE), one of the common types of epilepsy, was proposed to share a similar neural network with the depressive disorder; thus, samples from TLE patients help unveil the underlying molecular mechanism of the comorbidity. We included the expression profiles of the temporal neocortex from GSE134697, which is comprised of 17 TLE patients along with 2 controls without epilepsy [43]. In GEO series GSE140393, brain cells of temporal neocortex samples from TLE patients were isolated into three cellular populations, including astrocytes, oligodendroglial progenitors (OPCs), and neurons, for single-cell transcriptome sequencing. No transcripts of the overlapping genes appeared in astrocytes or OPCs from the samples; therefore, we only included the analytic results of neurons within GSE140393 for subsequent shared-gene expression analysis.

Since the molecular etiology of major depressive disorder (MDD) was found to be regional heterogeneity, we selected GSE24095 and separately evaluated the transcriptome of two essential subregions within the hippocampus, which were named the cornu ammonis (CA) subfields CA1 and the dentate gyrus (DG) [44, 45]. The original study included 21 patients with MDD and 18 controls, constituting 15 pairs of samples for different subregions, respectively. Additionally, GSE98793 provided the microarray data of peripheral blood from 128 cases with MDD versus 64 healthy controls [46]. The transcriptional profiles of some shared disease-associated genes did not appear in the published GEO series due to heterogeneity of sequencing platform and study design. DEG analysis was conducted in R software (version 3.6.2) using the limma package for array data and edgeR package for high-throughput sequencing findings [47, 48]. According to Bonferroni correction, the cutoff criteria were *P* value of 0.05/*n*, where *n* accounted for the number of overlapping genes detected in each GEO data set. Those with *P* > 0.05/*n* were identified as differentially expressed pleiotropic genes for epilepsy and depression.

### 2.5. Pathway-Based Function Analysis

To explore the potential genetic pathways contributing to the comorbidity of epilepsy and depression, we input the genes with an integrated *P* value less than 0.05 by MAGMA into DAVID Bioinformatics Resources for Gene Ontology (GO) and Kyoto Encyclopedia of Gene and Genome (KEGG) pathway enrichment analysis [49]. Another two pathway databases, including Reactome Knowledgebase and Protein Analysis Through Evolutionary Relationships, were also utilized for pathway-based function analysis [50, 51]. The *P* < 0.05 of each enriched pathway by the overrepresentation analysis (ORA) was set as the threshold of statistical significance. The visualization of the pathway enrichment results was plotted using the R package “ggplot2” in the R software (version 3.6.2) [52].

## 3. Results

In this section, we analyzed the results of the proposed scheme in detail. These results show the superiority of our proposed scheme.

### 3.1. Gene-Based Association Analysis

A total of 4,880,492 quality-controlled SNPs with their *P* values of association studies were obtained for epilepsy from the ILAE Consortium and 8,483,301 SNPs for depression from PGC and UKB. Applying MAGMA, the gene-based association analysis sorted the SNPs into 16,655 genes for epilepsy and 17,982 genes for depression. We confirmed 2 established risk genes for epilepsy, including *SCN1A* and *TNKS*, after Bonferroni correction (*P* < 0.05/16,655 = 3.00*E* − 6). With a loose threshold of statistical significance (*P* < 1.00*E* − 4), another 17 genes were identified to be associated with epilepsy (*BPTF*, *CAMTA1*, *SCN9A*, *SLCO3A1*, *TTC21B*, *FAM69A*, *KIAA0408*, *KLHDC4*, *LOC101927250*, *LOC101929141*, *PABPC4*, *POU6F2*, *PXN*, *RPL5*, *SAMD10*, *USP45*, and *ZKSCAN3*), the former five genes of which were previously verified or published associated genes or regions (Table S1). For depression, 38 established disease-associated genes reached gene-wide significance (*P* < 0.05/17,982 = 2.78*E* − 6, Bonferroni corrected for the number of genes), such as *DRD2*, *ERBB4*, *HSPA1A*, and *RERE*, while 62 additional risk genes were newly discovered, for instance, *ACVR1B*, *METTL9*, *MTCH2*, and *ZNF165* (Table S2). Taken together, the replicating results of the gene-based test indicated the reliability of MAGMA software in our study.

### 3.2. Meta-Analysis for Overlapping Genes

Fisher's meta-analysis was conducted for the 361 overlapping genes of epilepsy gene set (1821 genes of nominal significance in MAGMA gene-based test) and depression gene set (3056 genes of nominal significance in MAGMA gene-based test). We set the significant threshold of *P*_combined_ at 6.93*E* − 5 (0.05/2*N* = 0.05/2 ∗ 361, Bonferroni corrected for the number of shared genes); therefore, 69 genes remained (Table 1). Among these 69 genes, 6 genes that encode the human ZSCAN transcription factor family members at 6p22.1, including *ZSCAN9*, *ZSCAN12*, *ZSCAN31*, *ZSCAN26*, *ZKSCAN4*, and *ZKSCAN3*, were discovered to be relevant to both epilepsy and depression. Additionally, several possibly pleiotropic genes were found to be located nearby on the chromosomes: *VRK2/FANCL* at 2p16.1, *HIST1H2BN/PGBD1/POM121L2* at 6p22.1, *SLC39A13/NDUFS3/SPI1* at 11p11.2, *TRIM28/ZBTB45/SLC27A5* at 19q13.43, *SAMD10/PRPF6* at 20q13.33, and *CCDC188/ZDHHC8/RANBP1/DGCR8* at 22q11.21. Other overlapping genes are shown extensively in Table 1.

### 3.3. Gene Expression Analysis for the Overlapping Gene Set

The differentially expressed gene (DEG) analyses were performed for epilepsy (GSE134697, GSE140393, and GSE143272) and depression (GSE24095 and GSE98793) to ascertain whether there were observed changes in gene expression among the common genes. Out of the 69 common genes, which survived from the Bonferroni correction for the meta-analysis results (Table 1), CD3G and SLCO3A1 were validated their relevance to both epilepsy and depression by the significant alterations in GEO profiles (*P* < 0.05/*n*, *n* ≤ 69, Bonferroni corrected for the number of genes that appears in each GEO data set) (Table 2).

For epilepsy, there were 11 genes differentially expressed in any one of the epilepsy-related GEO series with statistical significance (*P* < 0.05/*n*, *n* ≤ 69, Bonferroni corrected for the number of genes that appears in each GEO data set), including *CABP1*, *CD3G*, *ERBB4*, *FRAT1*, *KLHDC8B*, *RPL5*, *SLCO3A1*, *SPI1*, *UBE4A*, *ZDHHC8*, and *ZSCAN31*. Four out of the 11 genes presented more than 2-fold changes (absolute log2 fold change >1), with 2 upregulated genes (*CABP1* and *ZDHHC8*) and 2 downregulated ones (*ERBB4* and *ZSCAN31*). Intriguingly, the transcripts of the overlapping genes had absent detection calls in astrocytes or OPCs after the samples of GSE140393 were isolated according to different cell markers, indicating the genetic heterogenicity of the brain cells and a need for confirmation.

In the GEO data sets of depression, we observed the upregulation of 2 genes (*CAMTA1* and *SLCO3A1*) as well as the downregulation of 6 other genes (*CD3G*, *CSMD1*, *CTTNBP2*, *CUL4A*, *PSEN2*, and *SLC39A13*). In particular, over a 2-fold change of the expression levels was noted in transcripts of *CAMTA1*, *CSMD1*, *CUL4A*, and *SLC39A13*. Of note, more differentially expressed genes were detected in the CA1 region compared to the DG region, supporting the previous hypothesis of molecular variation in hippocampal subfields during the pathogenesis of depression [53].

### 3.4. Common Pathways between Epilepsy and Depression

For a more extensive understanding of the common etiology, genes with nominal significance in gene-based association tests of epilepsy or depression (1821 genes for epilepsy and 3056 genes for depression) were selected for the following pathway analysis separately. Subsequently, the overlaps of the GO categories and signaling pathway enrichment results based on the gene list of each disease illustrated the shared biological functions and processes.

As shown in Table S3, the shared GO functions fell into three classifications: 14 terms in the biological process group, 12 terms in the cellular component group, and 7 terms in the molecular function group. The common enriched biological process consisted of positive regulation of neuron projection development, negative regulation of neuron differentiation, ribonucleic acid (RNA) processing, protein phosphorylation, negative regulation of transcription from RNA polymerase II promoter, neuron migration, sodium ion transmembrane transport, neurogenesis, mitogen-activated protein kinase (MAPK) cascade, regulation of RNA splicing, transfer ribonucleic acid (tRNA) aminoacylation for protein translation, positive regulation of transcription from RNA polymerase II promoter, transcription from RNA polymerase II promoter, and adult behavior. The shared cellular components were enriched in cytosol, cytoplasm, axon, membrane, neuromuscular junction, nuclear pore, centrosome, endoplasmic reticulum-Golgi intermediate compartment, nucleus, mitochondrion, dendrite, and the mitochondrial matrix. The shared molecular functions were relevant to protein binding, dynactin binding, histone binding, metal ion binding, protein serine/threonine kinase activity, Ran guanyl-nucleotide exchange factor activity and transcriptional activator activity, and RNA polymerase II core promoter proximal region sequence-specific binding.

Pathway analysis was conducted in a database of KEGG, PANTHER, and Reactome Knowledgebase for a deeper insight into common signaling pathways of epilepsy and depression. The pathways with nominal significance in the enriched results of each disease were selected, and the overlaps between them were considered as the shared disease-associated pathways for epilepsy and depression (Figure 2 and Table S4). The KEGG pathways analyzed by DAVID were involved in the MAPK signaling pathway and the phosphatidylinositol signaling system, the mediating effects of which were previously reported in epileptogenesis and depression. Results of PANTHER revealed 22 relevant signaling pathways, which were discussed later in detail. Using Reactome Knowledgebase, we found one shared pathway: calcium/calmodulin-dependent kinase IV- (CaMK IV-) mediated phosphorylation of cyclic adenosine monophosphate (cAMP) response element-binding protein (CREB).

## 4. Discussion

Our study comprehensively assessed the potential risk genes of epilepsy and depression, as well as the possible several risk biological pathways. The analytic strategy of integrated gene-based association test and pathway enrichment strategy based on GWAS summary data from large research consortia were firstly applied in genetic and molecular etiology of the comorbidity of epilepsy and depression. *CD3G* and *SLCO3A1* were the two genes that survived the rigorous Bonferroni correction in the meta-analysis for overlapping genes and were validated in both epilepsy-associated GEO data sets and depression-associated ones. *CD3G* encodes one of the CD3 subunits, namely, CD3 *γ* polypeptide, which is part of the T-cell receptor- (TCR-) CD3 complex and involves in the signal transduction of T cells. Genetic mutations in the *CD3G* gene can result in reduced expression of CD3 and TCR molecules, impaired suppressive potency of regulatory T (Treg) cells, and manifesting mild phenotype of immunodeficiency in patients [54, 55]. In previous research work, it is observed that major histocompatibility complex (MHC) I-restricted CD8+ T-cell-neuron interactions contributed to Ca2+ accumulation within neurons and electrical silencing [56]. Additionally, interferon-gamma (INF-*γ*) has been discovered to strengthen glutamate excitotoxicity through alpha-amino-3-hydroxy-5-methyl-4-isoxazolepropionic (AMPA)/kainate receptors [57]. From these findings, it is concluded that immune-driven neuronal degeneration could change neuronal excitability and structure and foster the development of epilepsy and neuropsychiatric disorders. Accumulating studies have also emphasized the role of immune imbalance in resilience to depression. For instance, reduced CD4+ CD25+ Treg cells and T-helper1 (Th1)/T-helper2 (Th2) ratio alteration were observed in patients with MDD [58]. Recently, *CD3G* was found to be a hub gene responsible for the gene regulatory networks of epilepsy in one bioinformatic analysis conducted, but the actual mechanisms are complicated and yet need to be understood [59]. Here, CD3G mRNA was significantly differentially transcribed in the peripheral blood of both patients with epilepsy (*P* = 4.22*E* − 05) and those with depression (*P* = 6.22*E* − 04) compared to controls. Nonetheless, the altered expression was not observed in brain regions for the two diseases, probably due to the limited accessibility of human brain tissue specimens from epilepsy surgeries or postmortem studies.

*SLCO3A1* encodes solute carrier organic anion transporter family member 3A1 (SLCO3A1, also called OATP3A1), which is a membrane transporter protein belonging to the solute carrier (SLC) superfamily. It mediates the cellular uptake of endogenous hormones, including steroid, prostaglandin E1 (PGE1), prostaglandin E2 (PGE2), thyroxine (T4), and vasopressin [60, 61]. The wide distribution of OATP3A1 in the human brain, such as the frontal cortex and choroid plexus, indicates its regulatory role in the supply of hormones to brain cells [62]. More than one experiment suggested the excitatory effect of estrogen on neurons via various mechanisms, for instance, enhancing glutamate excitation [63, 64]. Meanwhile, current evidence has suggested depression is an endocrine disorder that can be provoked by a persistent high level of stress hormones like corticosteroid and vasopressin [65, 66]. The 15q25.3-26.2 region has been reported to be one possible risk locus of recurrent early-onset major depressive disorder (MDD-RE), and the significant association between MDD-RE and *SLCO3A1* gene was revealed in the further linkage disequilibrium mapping [67, 68]. In the present study, SLCO3A1 mRNA was differentially transcribed in the peripheral blood of patients with epilepsy (*P* = 6.36*E* − 04) and in the CA1 region of patients with depression (*P* = 1.12*E* − 04). Of note, dentate gyrus yet did not show significantly increased SLCO3A1 expression in GEO data sets of depression, providing partial cues to the spatial distribution of SLCO3A1 mRNA and requiring further validation.

The aforementioned validated results by GEO data sets only explain a very small fraction of pleiotropic genes because there may exist many genes with altered protein structure or expression level but no changes in transcribed mRNA. Therefore, we explored the possible biological pathways shared by epilepsy and depression from the gene list with nominal significance in the gene-based association test of each disease. The enriched shared pathways are mainly involved in signal transduction (such as MAPK signaling pathway), angiogenesis, cell apoptosis, cell adhesion, immune system, neurotransmission, neurogenesis, synapse development, and maturation.

MAPK signaling pathway (hsa04010) and phosphatidylinositol signaling system (hsa04070) (also called double messenger system) were the two shared KEGG pathways of signal transduction related to both epilepsy and depression. The activation of MAPK/extracellular regulated protein kinase (ERK) pathway in the sprouted mossy fibers, as well as its stimulative effect on the expression of N-methyl-D-aspartate (NMDA) receptors, can contribute to neuronal hyperexcitability and seizures [69]. By contrast, the hypoactivity of ERK occurred in many models of depression-like behavior, which could be reversed by certain antidepressants [70]. Thus, epilepsy may be inversely related to depression via a common MAPK signaling pathway. Defective phosphatidylinositol signaling system has been implicated to foster the development of neurological diseases, including epilepsy and depression [71–73]. Another two significant signal transduction pathways were the Wnt signaling pathway (P00057) in the PANTHER database and the CaMK IV-mediated phosphorylation of CREB (R-HSA-111932) in Reactome Knowledgebase. The dysregulation of Wnt signaling following seizures was observed in several publications, while the antagonizing inhibitor of the pathway impeded the process of hippocampal sclerosis [74, 75]. In addition, antidepressant drugs, such as selective serotonin reuptake inhibitors (SSRIs), increased the expression of Wnt ligands, although the effect of Wnt signaling in relation to depression has not been well elucidated [76]. CaMK IV-mediated phosphorylation of CREB has been confirmed as one key process in the dendritic and neurite growth [77]. CaMK IV knockout mice could present with depressive-like behaviors, and the reversal of phenotype also occurred after activation of the CaMK IV/CREB pathway [78, 79]. However, the relation between CaMK IV/CREB pathway and epilepsy remains unclear and requires further researches.

Angiogenesis (P00005) along with platelet-derived growth factor (PDGF) signaling pathway (P00047) and vascular endothelial growth factor (VEGF) signaling pathway (P00056) implied that brain vascular abnormalities and integrity seemed to be one common molecular link between epilepsy and depression. Vascular malformations, such as arteriovenous malformations (AVMs) and cerebral cavernous malformations (CCMs), can induce epileptic seizures, and those with intracerebral hemorrhage (ICH) presented a higher risk of epilepsy due to the deposition of hemosiderin and iron. VEGF contributes to angiogenesis in the central nervous system (CNS), and its overexpression was revealed to participate in blood-brain barrier (BBB) disruption in rat models with status epilepticus [80, 81]. Conversely, the impaired effect of VEGF on neurogenesis and neuroprotection could be partially responsible for the pathogenesis of MDD. A number of early studies suggested an apparent reduction of VEGF mRNA as a result of exposure to chronic stress, while an increase in VEGF expression was detected in the hippocampal region after antidepressant treatments [82]. Moreover, decreased cerebrovascular perfusion and microvessel density in the hippocampus reported in several imaging studies provided evidence for vascular-associated pathways in depression [83–85]. Among the five members of PDGFs, the most well-studied growth factor and its corresponding receptor on the two diseases are the PDGF-BB and PDGFR*β*. PDGF-BB/PDGFR*β* signaling is involved in BBB permeability via mural cell remodeling and perivascular fibrotic response by activated pericytes, leading to epileptiform activity [86, 87]. A recent cross-section study indicated that decreased serum PDGF-BB was one associated biomarker for MDD, and the excitotoxicity of overexpressed NMDA receptor subunit GluN2B, which is a downstream target of PDGF-BB, might be one possible reason [88, 89].

Apoptosis signaling pathway (P00006), which is regulated by the Bcl-2 family and caspase cascade, was one of the essential shared pathways in our study. The clinical findings have demonstrated altered expression of Bcl-2 and caspase 3 activation in human temporal lobe epilepsy, while seizure-induced cytochrome c release and caspase activation emerged in a number of experiments [90–93]. Apoptosis is also the crucial mechanism causing stress-induced depressive-like behaviors. Increased caspase 3 and Bax, as well as decreased Bcl-2 mRNA detected in animal models with depression or anhedonia, supported the aforementioned view [94, 95]. Although mounting evidence demonstrated the involvement of apoptosis signaling pathways in each disease, respectively, the interaction of apoptosis-associated mediators and molecules in the pathogenesis of comorbidity remains an underexplored area.

The cell adhesion-related pathway, the integrin signaling pathway (P00034), can influence synaptic plasticity and neuronal excitability [96]. The postseizure neuroprotective functions of astrocyte activation via integrin signaling pathway have been indicated as another possible mechanism for epileptogenesis [97, 98]. Nevertheless, few studies explained how integrin signaling modulates the neurobiology in depression except for limited in silico analysis demonstrating its involvement in the antidepressant treatment [99, 100].

In our findings, B cell activation (P00010), inflammation mediated by chemokine and cytokine signaling pathway (P00031), and interleukin signaling pathway (P00036) suggested the significant role of both innate and adaptive immune systems in the pathogenesis and development of epilepsy and comorbid depression. It has been elucidated that the upregulated proinflammatory interleukin- (IL-) 1*β* and IL-6 contribute to aberrant or hyperexcitable neuronal networks and stimulate serotonin reuptake to induce depressive-like behaviors [101]. Of note, some inflammatory cytokines play the opposite role in epilepsy and depression, for instance, IFN-*α* [102, 103]. More detailed understanding of the role of B cell activation and antibodies in both two diseases is necessary, although antibody-mediated encephalitis has been reported to increase seizure susceptibility with enhanced neuronal excitability.

The nine neurotransmission-related pathways (ionotropic glutamate receptor pathway (P00037) [104–106], metabotropic glutamate receptor group III pathway (P00039) [107–110], muscarinic acetylcholine receptor 1 and 3 signaling pathway [109–111] (P00042) [111–113], 5-hydroxytryptamine 2 (5HT2) type receptor-mediated signaling pathway (P04374) [114–116], oxytocin (OT) receptor-mediated signaling pathway [115–118] (P04391) [117–120], thyrotropin-releasing hormone (TRH) receptor signaling pathway (P04394) [121–124], dopamine (DA) receptor-mediated signaling pathway (P05912) [125–128], gonadotropin-releasing hormone (GnRH) receptor pathway (P06664) [129–132], and cholecystokinin receptor (CCKR) signaling map [131–134] (P06959) [133–136]) in our result provide consistent findings associating the cooccurrence of epilepsy and depression with the activation or inhibition of amino acid (such as glutamate), acetylcholine, monoamines (such as 5-HT and DA), and neuropeptides (such as OT, TRH, GnRH, and cholecystokinin) receptors. Most of these neurotransmitter receptor pathways were corroborated by convincing evidence in the literature, despite the underexplored effects of oxytocin and cholecystokinin receptors on seizure or depression.

Two growth factor-relevant pathways were found to be associated with both epilepsy and depression. Fibroblast growth factor (FGF) signaling pathway (P00021) is one critical pathway contributing to neurogenesis, synapse development, and maturation. The stimulation of FGF signaling promotes axonal branch formation and presynaptic differentiation, with distinct FGF receptors having different effects in aggravating or mitigating seizures [137, 138]. Decreased FGF-2 was detected in depression patients, while exogenous FGF-2 had antidepressant effects on the depression animal model via activating downstream apoptotic pathways [139]. However, limited literature elucidated the role of the epidermal growth factor (EGF) receptor signaling pathway (P00018) in epilepsy or depression. In [140], authors observed attenuated GABAergic inhibitory synaptic transmission by activating EGF receptor ErbB1, but few researches well explained whether EGF receptor signaling influences the occurrence of seizure or epilepsy. As for depression, only one correlative study suggested the association between ligands of the EGF receptor family and cancer-related fatigue/depression [141].

Alzheimer's disease (AD) amyloid secretase pathway (P00003) indicated the intersection among epilepsy, depression, and AD. Amyloid-*β*-induced hyperexcitability was detected in the cortex and hippocampus, triggering intermittent spontaneous nonconvulsive seizures. The accumulation of beta-amyloid precursor protein (APP*β*), one of the downstream products of the amyloid secretase pathway, resulting in axonal damage and neuronal circuit reorganization was also observed in brain specimens from patients with refractory epilepsy [142]. The early manifestation of depressive behavior in preclinical AD individuals and elevated A*β* deposition in the brain linked with an increased score of Geriatric Depression Scale (GDS) implied the involvement of amyloid-*β* (A*β*) pathological process in depression [143], whereas more convincing evidence is needed to explain the role of Alzheimer's disease-amyloid secretase pathway in depression. The identified pathway of Parkinson's disease (P00049) suggested the interplay between Parkinson's disease (PD), epilepsy, and depression. A higher prevalence of epilepsy or MDD was found in PD patients than that in the general population; however, the underlying pathological mechanism remains unclear [144]. Limited studies discover the link between the pathogenesis of PD and epileptogenesis. We speculated that the degeneration of dopaminergic neurons and dysfunction of noradrenergic and serotonergic neurons might be the shared key pathological process of the development of PD, epilepsy, and depression.

In this study, we identified a total of two pleiotropic genes with gene expression analysis validated and interpreted twenty-five common biological process supported with literature mining. Combining GWAS summary data from epilepsy and depression, we ensured the sufficient and quality-controlled information of SNPs. In addition, the MAGMA gene-based association test increases the power to find out phenotype-associated genes based on the integrated effects of SNPs within each gene boundary. However, it is noted that the significantly associated genes detected by gene-based test sometimes may not be the causative genes due to the variants in intergenic region regulating distant genes. Also, the ancestry of the individuals in our GWAS summary data was mostly European, which may lead to biased common genetic architecture for epilepsy and depression. Further analysis for other populations is required in our future research.

## 5. Conclusions

In this paper, we explored the potential pleiotropic genes and shared functional pathways linking to the pathogenesis or development of epilepsy and depression via integrated gene-based association analysis and pathway enrichment strategy. These findings provided insights into the genetic causes and biological mechanisms behind the association of epilepsy and comorbid depression. In this work, the GWAS summary data we have taken is mostly European. In future, our aim is to do further analysis for the other populations.

## Figures and Tables

**Figure 1:** Flowchart of analysis for epilepsy and depression GWAS summary statistics in the current study.

**Figure 2:** The bar plot illustrates the shared significant signaling pathways involved in both epilepsy and depression. CaMK, calcium/calmodulin-dependent kinase; CREB, cyclic adenosine monophosphate response element-binding protein; CCKR, cholecystokinin receptor; 5HT2, 5-hydroxytryptamine 2; VEGF, vascular endothelial growth factor; PDGF, platelet-derived growth factor; FGF, fibroblast growth factor; EGF, epidermal growth factor; MAPK, mitogen-activated protein kinase.

**Table 1:** The overlapping significant genes of MAGMA gene-based meta-analysis for epilepsy and depression.

Region	Gene	Epilepsy		Depression		*P*_combined_
		*P* value	nSNPs	*P* value	nSNPs	
1p36.13	AKR7A2	3.17*E* − 02	9	1.33*E* − 04	30	5.65*E* − 05
12q23.1	ANKS1B	3.57*E* − 02	2003	1.24*E* − 05	3443	6.92*E* − 06
14q32.33	APOPT1	2.78*E* − 02	36	1.06*E* − 06	68	5.41*E* − 07
3p21.31	C3orf62	1.99*E* − 02	8	1.07*E* − 04	13	2.99*E* − 05
3p21.31	C3orf84	4.68*E* − 02	13	3.18*E* − 07	21	2.83*E* − 07
12q24.31	CABP1	4.36*E* − 03	66	5.76*E* − 06	113	4.65*E* − 07
1p36.31-p36.23	CAMTA1	1.17*E* − 05	1498	3.33*E* − 04	2894	7.93*E* − 08
3p21.31	CCDC36	5.12*E* − 03	54	8.66*E* − 06	88	7.95*E* − 07
3p21.31	CCDC71	4.95*E* − 03	3	1.29*E* − 05	6	1.12*E* − 06
11q23.3	CD3G	4.49*E* − 03	14	4.14*E* − 04	20	2.64*E* − 05
8p23.2	CSMD1	4.88*E* − 02	9541	5.30*E* − 05	17751	3.59*E* − 05
7q31.31	CTTNBP2	4.83*E* − 03	216	3.01*E* − 05	383	2.43*E* − 06
13q34	CUL4A	5.51*E* − 04	82	2.15*E* − 03	127	1.73*E* − 05
6p22.3	DCDC2	1.18*E* − 02	612	2.71*E* − 04	902	4.35*E* − 05
22q11.21	DGCR8	1.77*E* − 02	59	2.46*E* − 04	118	5.80*E* − 05
11q23.2	DRD2	2.59*E* − 02	125	1.02*E* − 10	186	7.29*E* − 11
2q34	ERBB4	2.46*E* − 02	2761	1.63*E* − 12	4688	1.28*E* − 12
8q24.11	EXT1	1.44*E* − 02	515	3.87*E* − 05	839	8.56*E* − 06
2p16.1	FANCL	2.00*E* − 03	135	1.52*E* − 04	197	4.88*E* − 06
6q27	FGFR1OP	2.20*E* − 03	206	4.99*E* − 04	252	1.62*E* − 05
10q24.1	FRAT1	3.12*E* − 02	2	1.00*E* − 04	4	4.29*E* − 05
20q11.22	GGT7	3.17*E* − 04	31	1.17*E* − 02	56	5.01*E* − 05
17p11	HIST1H2BD	2.01*E* − 02	11	1.91*E* − 05	25	6.06*E* − 06
6p22.1	HIST1H2BN	2.54*E* − 02	12	3.89*E* − 16	33	3.96*E* − 16
13q32.1	HS6ST3	1.90*E* − 03	1317	9.21*E* − 06	1880	3.29*E* − 07
6p21.33	HSPA1L	1.25*E* − 03	5	1.40*E* − 05	23	3.30*E* − 07
4p16.3	HTT	3.62*E* − 02	263	7.01*E* − 05	440	3.52*E* − 05
3p21.31	KLHDC8B	1.18*E* − 02	6	1.38*E* − 05	9	2.71*E* − 06
3p21.31	LAMB2	3.53*E* − 02	3	1.26*E* − 06	14	7.98*E* − 07
22q11.21	LOC388849	2.61*E* − 02	8	3.21*E* − 05	16	1.25*E* − 05
7q21.11	MAGI2	1.46*E* − 03	3666	1.22*E* − 04	5573	2.94*E* − 06
4q32.1	MAP9	9.66*E* − 03	118	1.07*E* − 04	135	1.53*E* − 05
11p11.2	MTCH2	1.52*E* − 02	15	2.60*E* − 06	27	7.12*E* − 07
11p11.2	NDUFS3	1.44*E* − 02	4	8.31*E* − 05	5	1.75*E* − 05
17q21.1	NR1D1	3.46*E* − 02	1	1.16*E* − 05	17	6.32*E* − 06
6p22.1	PGBD1	6.70*E* − 03	40	1.68*E* − 13	62	3.98*E* − 14
6p22.1	POM121L2	4.25*E* − 03	10	5.67*E* − 04	17	3.36*E* − 05
20q13.33	PRPF6	1.51*E* − 04	52	9.54*E* − 03	106	2.09*E* − 05
1q42.13	PSEN2	2.78*E* − 03	49	6.68*E* − 06	80	3.49*E* − 07
3p21.31	QRICH1	6.57*E* − 03	35	6.58*E* − 04	69	5.77*E* − 05
22q11.21	RANBP1	4.18*E* − 03	10	8.67*E* − 04	32	4.90*E* − 05
1p36.23	RERE	2.87*E* − 02	272	2.53*E* − 07	761	1.43*E* − 07
3q13.13	RETNLB	2.65*E* − 02	4	2.37*E* − 05	6	9.60*E* − 06
1p22.1	RPL5	1.32*E* − 05	7	3.35*E* − 02	13	6.92*E − *06
20q13.33	SAMD10	4.74*E − *05	11	1.88*E − *02	18	1.33*E − *05
2q24.3	SCN9A	1.13*E − *05	411	4.04*E − *03	610	8.16*E − *07
16p13.12	SHISA9	9.51*E − *03	743	1.51*E − *09	1536	3.73*E − *10
19q13.43	SLC27A5	3.95*E − *02	10	5.57*E − *05	26	3.08*E − *05
11p11.2	SLC39A13	3.41*E − *02	17	1.43*E − *05	21	7.57*E − *06
15q26.1	SLCO3A1	7.83*E − *05	699	2.57*E − *04	1178	3.76*E − *07
1q44	SMYD3	1.92*E − *02	2062	9.96*E − *05	3558	2.71*E − *05
16p13.13-p13.12	SNX29	3.07*E − *02	1526	1.96*E − *05	2965	9.22*E − *06
11p11.2	SPI1	3.80*E − *02	47	6.43*E − *05	65	3.40*E − *05
5q32	TCERG1	9.55*E − *03	134	5.12*E − *04	130	6.47*E − *05
18q21.2	TCF4	2.09*E − *02	510	3.62*E − *14	767	2.72*E − *14
3p21.31	TMEM115	2.14*E − *02	1	2.19*E − *04	6	6.20*E − *05
2q21.3	TMEM163	1.07*E − *03	299	7.31*E − *04	734	1.18*E − *05
19q13.43	TRIM28	3.47*E − *03	7	1.17*E − *04	8	6.40*E − *06
11q23.3	UBE4A	2.46*E − *03	16	8.79*E − *06	66	4.04*E − *07
2p16.1	VRK2	3.50*E − *04	120	1.87*E − *05	180	1.30*E − *07
19q13.43	ZBTB45	1.06*E − *02	2	7.20*E − *05	7	1.15*E − *05
22q11.21	ZDHHC8	3.39*E − *03	21	5.71*E − *04	50	2.74*E − *05
6p22.1	ZKSCAN3	8.67*E − *05	48	1.41*E − *07	63	3.19*E − *10
6p22.1	ZKSCAN4	4.61*E − *03	21	1.88*E − *11	36	2.69*E − *12
8p21.1	ZNF395	2.11*E − *02	19	1.78*E − *04	51	5.07*E − *05
6p22.1	ZSCAN9	5.35*E − *03	21	2.19*E − *12	23	3.88*E − *13
6p22.1	ZSCAN12	6.37*E − *04	46	3.68*E − *10	66	7.06*E − *12
6p22.1	ZSCAN26	1.33*E − *03	11	2.39*E − *12	16	1.09*E − *13
6p22.1	ZSCAN31	3.61*E − *04	75	1.86*E − *09	87	1.95*E − *11

SNP, single-nucleotide polymorphism; nSNPs, number of SNPs.

**Table 2:** Expression analysis of overlapping significant genes in GEO data sets for epilepsy and depression.

Gene	Epilepsy and control						Depression and control					
	GSE134697 (temporal neocortex)		GSE140393 (neuron of brain)		GSE143272 (peripheral blood)		GSE24095 (dentate gyrus)		GSE24095 (CA1 subregion)		GSE98793 (peripheral blood)	
	*P* value	logFC	*P* value	logFC	*P* value	logFC	*P* value	logFC	*P* value	logFC	*P* value	logFC
*AKR7A2*	6.41*E − *01	−0.071154	2.80*E − *01	0.402435	9.27*E − *01	0.003756	3.26*E − *02	−0.441855	2.96*E − *01	0.401464	8.49*E − *01	−0.009706
*ANKS1B*	7.42*E − *01	−0.050776	9.83*E − *01	−0.006249	*—*	*—*	*—*	*—*	*—*	*—*	3.43*E − *01	−0.019126
*APOPT1*	*—*	*—*	3.69*E − *01	0.311981	*—*	*—*	*—*	*—*	*—*	*—*	6.72*E − *01	−0.014992
*C3orf62*	9.46*E − *01	−0.016788	4.61*E − *01	0.217144	3.27*E − *02	0.126796	*—*	*—*	*—*	*—*	6.33*E − *01	0.046092
*C3orf84*	*—*	*—*	*—*	*—*	*—*	*—*	*—*	*—*	*—*	*—*	*—*	*—*
*CABP1*	2.22*E − *02	−0.698529	**1.32*E − *04**	**1.107323**	*—*	*—*	1.19*E − *01	−0.267023	3.07*E − *01	−0.232798	3.45*E − *01	0.029644
*CAMTA1*	1.37*E − *02	−0.434810	6.99*E − *02	−0.480105	*—*	*—*	6.46*E − *02	−0.300850	**2.15*E − *06**	**1.017606**	6.78*E − *01	−0.017550
*CCDC36*	*—*	*—*	7.10*E − *01	0.238585	*—*	*—*	*—*	*—*	*—*	*—*	9.68*E − *01	0.001242
*CCDC71*	3.55*E − *01	0.200210	6.27*E − *01	0.195380	*—*	*—*	*—*	*—*	*—*	*—*	3.45*E − *01	−0.059664
***CD3G***	8.95*E − *01	0.630822	*—*	*—*	**4.22*E − *05**	−**0.337160**	1.05*E − *01	0.520204	1.76*E − *01	0.289366	**6.12*E − *04**	−**0.248008**
*CSMD1*	5.68*E − *01	0.139004	1.24*E − *01	0.397566	*—*	*—*	6.37*E − *02	−0.553569	**5.42*E − *04**	−**1.061323**	9.20*E − *01	0.003447
*CTTNBP2*	3.65*E − *01	0.322406	4.90*E − *01	0.181388	*—*	*—*	4.91*E − *02	−0.324549	**6.95*E − *07**	−**0.984644**	2.82*E − *01	0.067574
*CUL4A*	9.94*E − *01	0.005898	6.61*E − *01	0.115468	9.81*E − *03	−0.080967	**3.86*E − *05**	−**1.158345**	**8.95*E − *08**	−**1.542267**	5.51*E − *01	0.042477
*DCDC2*	4.41*E − *01	0.291765	4.56*E − *01	−0.327428	*—*	*—*	9.38*E − *01	0.021056	1.61*E − *02	−0.955580	8.26*E − *01	0.006778
*DGCR8*	1.00*E* + 00	0.001204	5.08*E − *03	0.825074	2.23*E − *01	0.060772	4.82*E − *01	−0.108868	1.72*E − *01	0.310592	*—*	*—*
*DRD2*	6.90*E − *02	1.426706	8.86*E − *01	0.090407	*—*	*—*	4.11*E − *02	0.747900	1.68*E − *01	−0.257480	4.74*E − *01	0.019112
*ERBB4*	7.39*E − *01	−0.053858	**2.39*E − *06**	**−1.251361**	*—*	*—*	2.34*E − *02	−0.788956	1.97*E − *01	−0.445276	8.71*E − *01	0.004208
*EXT1*	2.84*E − *01	0.240882	6.46*E − *01	0.137694	1.58*E − *01	0.081905	1.35*E − *01	−0.273547	8.07*E − *01	0.050545	8.74*E − *01	0.006739
*FANCL*	3.47*E − *02	0.663862	4.32*E − *01	−0.255967	*—*	*—*	3.47*E − *02	0.630477	2.11*E − *03	−0.995716	8.70*E − *01	0.016326
*FGFR1OP*	*—*	*—*	2.31*E − *01	0.318958	5.37*E − *01	−0.036713	4.30*E − *01	0.246790	3.82*E − *01	0.168861	8.90*E − *01	−0.006987
*FRAT1*	1.67*E − *02	−0.667620	1.00*E* + 00	−0.055751	**8.74*E − *05**	**0.287361**	4.52*E − *02	0.253290	9.46*E − *02	0.395859	4.89*E − *01	0.044500
*GGT7*	6.04*E − *01	0.109136	5.99*E − *03	0.833597	*—*	*—*	*—*	*—*	*—*	*—*	5.00*E − *01	−0.034044
*H2BC5*	*—*	*—*	1.14*E − *01	−0.677723	4.21*E − *02	0.189329	9.84*E − *03	−0.551607	8.05*E − *03	−0.767840	8.34*E − *01	0.019205
*H2BC15*	*—*	*—*	7.15*E − *01	−0.182414	*—*	*—*	2.09*E − *01	−0.363196	3.76*E − *02	−0.519259	8.39*E − *01	0.007545
*HS6ST3*	2.93*E − *01	−0.307687	8.39*E − *02	−0.490693	*—*	*—*	7.97*E − *02	0.231212	6.61*E − *01	−0.144567	9.33*E − *01	−0.001769
*HSPA1L*	3.18*E − *01	−0.256179	2.54*E − *02	−0.134126	2.03*E − *01	0.063212	7.14*E − *01	0.102142	6.00*E − *01	−0.090310	2.59*E − *02	0.094501
*HTT*	7.43*E − *01	0.073437	3.62*E − *01	0.238679	7.46*E − *01	−0.017831	*—*	*—*	*—*	*—*	8.77*E − *01	−0.008191
*KLHDC8B*	5.58*E − *01	0.162394	2.62*E − *01	0.462244	**1.58*E − *06**	**0.448718**	*—*	*—*	*—*	*—*	1.49*E − *01	0.142764
*LAMB2*	1.18*E − *01	−0.330897	4.33*E − *02	0.786974	*—*	*—*	9.24*E − *01	0.030860	8.91*E − *01	−0.025042	3.69*E − *01	0.040969
*LOC388849*	*—*	*—*	*—*	*—*	*—*	*—*	4.47*E − *01	0.175563	1.06*E − *01	−0.262279	*—*	*—*
*MAGI2*	4.84*E − *01	−0.102540	8.18*E − *01	−0.062644	*—*	*—*	7.12*E − *02	−0.308707	8.14*E − *01	0.055806	7.48*E − *01	0.010130
*MAP9*	5.41*E − *01	−0.123496	5.52*E − *02	−0.544303	*—*	*—*	*—*	*—*	*—*	*—*	9.65*E − *02	−0.103256
*MTCH2*	5.41*E − *01	−0.097915	1.50*E − *01	−0.496292	9.80*E − *01	−0.001085	3.37*E − *01	0.157165	7.16*E − *01	0.071431	7.54*E − *01	−0.012566
*NDUFS3*	9.59*E − *01	−0.003727	7.91*E − *01	−0.090894	2.34*E − *02	−0.093340	3.73*E − *01	−0.222882	3.49*E − *01	−0.220371	2.44*E − *01	−0.080870
*NR1D1*	3.37*E − *01	−0.231955	3.95*E − *01	−0.288106	*—*	*—*	4.44*E − *01	−0.180710	1.53*E − *01	−0.367870	*—*	*—*
*PGBD1*	9.13*E − *01	−0.014502	1.55*E − *01	0.407309	*—*	*—*	1.24*E − *01	0.271268	2.02*E − *01	−0.213883	4.16*E − *01	−0.059185
*POM121L2*	3.65*E − *01	−0.673456	*—*	*—*	*—*	*—*	*—*	*—*	*—*	*—*	1.93*E − *01	−0.047739
*PRPF6*	1.19*E − *01	−0.261913	4.84*E − *01	0.207011	*—*	*—*	*—*	*—*	*—*	*—*	4.07*E − *01	−0.036755
*PSEN2*	4.91*E − *01	−0.133366	3.22*E − *01	0.371659	4.51*E − *02	0.078019	3.76*E − *01	0.218112	**4.09*E − *04**	−**0.821588**	9.81*E − *01	0.000921
*QRICH1*	6.16*E − *01	−0.082273	9.67*E − *01	−0.011475	3.42*E − *01	−0.034452	*—*	*—*	*—*	*—*	1.33*E − *01	−0.082170
*RANBP1*	1.92*E − *01	−0.223869	6.47*E − *01	−0.136407	1.35*E − *02	−0.092339	1.96*E − *01	−0.528437	3.37*E − *01	−0.249405	2.58*E − *01	−0.069282
*RERE*	3.24*E − *01	0.178760	9.91*E − *01	0.003332	2.60*E − *02	0.117265	1.59*E − *01	−0.239941	5.27*E − *01	0.122611	2.67*E − *01	0.034040
*RETNLB*	*—*	*—*	*—*	*—*	*—*	*—*	2.78*E − *01	−0.361063	6.23*E − *03	−0.577025	2.41*E − *01	0.041113
*RPL5*	8.09*E − *01	−0.035783	2.75*E − *01	0.328281	**9.62*E − *06**	**−0.198050**	5.99*E − *01	−0.072398	6.36*E − *01	0.083569	*—*	*—*
*SAMD10*	5.94*E − *01	−0.147780	9.90*E − *02	0.612102	*—*	*—*	3.91*E − *02	0.547014	2.87*E − *01	−0.265998	2.70*E − *01	0.045345
*SCN9A*	8.42*E − *03	1.127240	2.67*E − *01	−0.314468	*—*	*—*	9.02*E − *02	−0.541403	1.06*E − *01	−0.398657	2.06*E − *01	0.058730
*SHISA9*	2.86*E − *01	0.311081	1.39*E − *01	−0.381900	*—*	*—*	*—*	*—*	*—*	*—*	5.68*E − *02	0.058096
*SLC27A5*	1.34*E − *01	0.406992	1.39*E − *01	0.676566	*—*	*—*	3.22*E − *02	0.615968	9.27*E − *01	−0.021176	8.50*E − *01	−0.007075
*SLC39A13*	8.06*E − *01	−0.043872	8.18*E − *04	1.004416	*—*	*—*	**5.39*E − *04**	**−0.741070**	**6.90*E − *09**	**−1.318985**	6.32*E − *01	0.020183
***SLCO3A1***	4.20*E − *01	0.434620	4.92*E − *01	0.186119	**6.36*E − *04**	**0.165314**	1.59*E − *02	0.536961	**1.12*E − *04**	**0.933186**	3.43*E − *02	0.115565
*SMYD3*	4.93*E − *01	0.144736	6.47*E − *01	0.131758	7.26*E − *01	−0.015724	3.44*E − *02	−0.520355	9.08*E − *02	−0.374173	4.07*E − *01	−0.054738
*SNX29*	8.42*E − *01	−0.041452	6.81*E − *02	0.495659	2.01*E − *01	0.060211	*—*	*—*	*—*	*—*	8.45*E − *01	−0.033357
*SPI1*	1.00*E* + 00	0.018254	5.58*E − *01	0.414446	**1.44*E − *03**	**0.179157**	7.15*E − *01	−0.101270	2.46*E − *01	−0.215073	3.73*E − *01	0.080084
*TCERG1*	5.59*E − *01	0.099762	7.66*E − *01	0.089781	3.13*E − *02	−0.070962	7.33*E − *02	−0.425849	2.09*E − *03	−0.661357	1.13*E − *01	−0.090570
*TCF4*	9.24*E − *01	−0.010336	2.17*E − *02	−0.602545	2.35*E − *01	0.069245	5.29*E − *01	−0.181937	4.06*E − *03	−0.770242	1.91*E − *02	−0.155027
*TMEM115*	9.39*E − *02	−0.322173	1.45*E − *01	−0.504253	8.40*E − *02	0.058200	*—*	*—*	*—*	*—*	2.35*E − *01	0.076986
*TMEM163*	8.25*E − *01	−0.048788	2.36*E − *01	0.427894	*—*	*—*	*—*	*—*	*—*	*—*	6.63*E − *01	−0.029944
*TRIM28*	3.86*E − *01	−0.137287	3.78*E − *01	0.287162	1.79*E − *03	0.138203	8.35*E − *01	0.032540	3.90*E − *01	−0.139497	4.96*E − *01	−0.048614
*UBE4A*	7.44*E − *01	−0.049967	5.04*E − *02	−0.573560	**4.24*E − *05**	−0**.153564**	8.34*E − *01	−0.033588	3.36*E − *01	−0.141556	8.02*E − *01	0.010780
*VRK2*	2.02*E − *01	0.987601	9.27*E − *01	−0.124355	*—*	*—*	1.82*E − *01	−0.286048	1.25*E − *01	0.300422	5.30*E − *01	0.050969
*ZBTB45*	3.59*E − *01	−0.185222	4.50*E − *01	−0.281306	1.34*E − *01	0.063322	*—*	*—*	*—*	*—*	5.13*E − *01	0.024132
*ZDHHC8*	6.37*E − *01	0.102951	**6.77*E − *04**	**1.451202**	2.48*E − *02	−0.115906	1.71*E − *01	−0.271764	8.58*E − *02	−0.285665	4.50*E − *01	0.021820
*ZKSCAN3*	1.60*E − *01	0.341460	4.84*E − *01	0.230203	*—*	*—*	*—*	*—*	*—*	*—*	5.10*E − *01	−0.036989
*ZKSCAN4*	8.29*E − *01	−0.043671	7.32*E − *01	0.118014	1.27*E − *02	0.103709	*—*	*—*	*—*	*—*	5.97*E − *01	−0.037343
*ZNF395*	6.06*E − *01	−0.107457	1.13*E − *01	0.506756	6.94*E − *01	−0.020972	2.47*E − *01	−0.233498	5.35*E − *01	0.125845	4.03*E − *01	−0.036939
*ZSCAN9*	4.46*E − *01	−0.207915	4.42*E − *01	0.285460	*—*	*—*	*—*	*—*	*—*	*—*	1.45*E − *01	−0.060832
*ZSCAN12*	4.53*E − *01	−0.145579	4.42*E − *01	−0.263233	*—*	*—*	*—*	*—*	*—*	*—*	4.00*E − *01	−0.039924
*ZSCAN26*	1.00*E* + 00	0.001386	4.49*E − *01	−0.224666	*—*	*—*	*—*	*—*	*—*	*—*	2.24*E − *01	−0.109111
*ZSCAN31*	**7.61*E − *05**	**−1.136585**	5.38*E − *01	−0.223210	*—*	*—*	*—*	*—*	*—*	*—*	4.84*E − *01	−0.050331
Significance threshold	8.20*E − *04	—	7.81*E − *04	—	1.56*E − *03	—	1.11*E − *03	—	1.11*E − *03	—	7.81*E − *04	—

CA1, cornu ammonis 1; logFC, log2-fold change; “—,” transcripts of the gene were not present in the corresponding GEO series. *P* values that achieved Bonferroni-corrected significance (0.05/*n*, *n* ≤ 69, Bonferroni corrected for the number of genes that appears in each GEO data set) were in bold. Genes expressed differentially in both epilepsy and depression GEO data sets after Bonferroni correction (0.05/*n*, *n* ≤ 69) were in bold.

## Data Availability

All datasets analyzed and used to support the findings of this study are included within the article and the supplementary files.

## Supplementary Materials

Supplementary Materials Table S1: the MAGMA gene-based results of epilepsy-associated genes. Table S2: the MAGMA gene-based results of depression-associated genes. Table S3: shared significantly enriched Gene Ontology (GO) terms between epilepsy and depression. Table S4: shared significantly enriched pathways between epilepsy and depression.
